# Acupuncture for Female Infertility: Discussion on Action Mechanism and Application

**DOI:** 10.1155/2022/3854117

**Published:** 2022-07-04

**Authors:** Jing-yu Xu, An-lan Zhao, Ping Xin, Jun-ze Geng, Bao-juan Wang, Tian Xia

**Affiliations:** ^1^First Teaching Hospital of Tianjin University of Traditional Chinese Medicine, Tianjin 300193, China; ^2^National Clinical Research Center for Chinese Medicine Acupuncture and Moxibustion, Tianjin 300193, China; ^3^Tianjin University of Traditional Chinese Medicine, Tianjin 300000, China

## Abstract

A higher incidence of female infertility has been reported with an unexpectedly early appearance in recent years. The female infertility treatment and application of assisted reproductive technology have recently gained immense interest from scientists. Many studies have discussed the beneficial effects of acupuncture on female infertility. With advancements in science and medical technology, acupuncture-related research has increased in investigating its effectiveness in treating female infertility. This review focuses on a compilation of research in recent years on acupuncture for female infertility treatment and the exploration of the underlying mechanism. For this purpose, literature was searched using various search engines like PubMed, Web of Science, and Google Scholar. The search was refined by only focusing on recent studies on acupuncture effectiveness and mechanism in female infertility and evaluating pregnancy outcomes.

## 1. Introduction

The reproduction cycle continued to work, but the primary focus was on arranging life commodities for the family in ancient times due to limited resources. The advancement in science and technology and the modernization of civilization led to an increase in the pace of people's lives. Their roles gradually diversified, which translated into an increase in the burden of responsibilities. Similarly, fertility seems no longer a “must” thing to ponder upon with the increasing enrichment of human spiritual culture. Although stupendous progress in human civilization is inevitable and cannot be segregated from spiritual beliefs, fertility problems demand attention.

An estimated 8 to 12% of couples of childbearing ages suffer infertility globally [1], and the incidence rate of female infertility is reported at 15% [2], making it the third primary disease after cancer and cardiovascular diseases. In addition, female infertility affects the women's psychological well-being and results in disturbed intrafamily harmony. With an increasing incidence rate of female infertility each year, it has become one of the urgent problems to be solved and has aroused the widespread concern of researchers. Infertility is a condition characterized by the failure to establish a clinical pregnancy after 12 months of regular unprotected sex [3]. Many factors, behaviors, and pathologies can hinder the pregnancy process and lead to infertility, except for artificial contraception [4].

Furthermore, increased age has also been regarded as one of the important contributing factors to female fertility [5]. The rate of female infertility incidence among younger women has increased in recent years [6]. Due to unhealthy lifestyles and environmental factors, the incidence of reproductive and endocrine diseases in female infertility is gradually growing, such as premature ovarian insufficiency (POI), polycystic ovary syndrome (PCOS), chronic endometritis (CE), and endometrial polyps [7]. They all hinder the occurrence of pregnancy from different nodes and lead to adverse pregnancy outcomes.

The recent increase in female infertility cases has also promoted the development and application of assisted reproductive technology, such as artificial insemination (AI), in vitro fertilization-embryo transfer (IVF-ET), and intracytoplasmic sperm injection (ICSI). However, the current success rate of AI and ET technology is reported to be 15% [8, 9] and 30 to 40% [10], respectively. Therefore, further improving the success rate of assisted reproductive technology is also the hotspot and focus of current research. The combined application of complementary and alternative medicine (CAM) and assisted reproductive technology may become a solution to improve the clinical pregnancy rate.

Acupuncture is an alternative auxiliary therapy that has existed for thousands of years and is widely used in clinical practice. There is much research evidence to support the therapeutic effect of acupuncture [11]. Traditional acupuncture is comprised of inserting a “needle” into specific parts (i.e., topically disinfected acupoints), followed by manipulation to enhance the sense of acupuncture after the needle enters the skin and reaches the site of action [12]. Later, with the progress of science and technology, to make the effect of acupuncture more obvious and lasting, a series of similar treatment methods have been derived, such as electroacupuncture (EA), acupoint catgut embedding (ACE), and transcutaneous electrical acupoint stimulation (TEAS) [13]. The working principle of EA, ACE, and TEAS is the same as that of traditional acupuncture, with only difference in the action parts and operating devices.

Being a novel subject, the development of assisted reproductive technology has gained much interest in recent years. The clinical efficacy of acupuncture in female infertility has undoubtedly aroused the interest of many reproductive doctors, and the research on acupuncture in female infertility has gradually increased, which provides a lot of evidence basis for the application of acupuncture in female infertility. This review summarizes the current application of acupuncture in treating female infertility. It further explores acupuncture's potential mechanism and application potential as an auxiliary and alternative therapy option for treating female infertility. This paper is also envisaged to promote research on acupuncture further and optimize the clinical treatment plan.

## 2. Causes of Female Infertility

Understanding female infertility requires prior knowledge and understanding of the pregnancy cycle. The pregnancy cycle starts with sperms entering the vagina and traveling upwards through the cervix into the uterus. The sperms then travel to fallopian tubes, meeting the ova and causing its fertilization. The fertilized egg follows the movement of cilia in the lining of the fallopian tube toward the uterine cavity. Once in the uterine cavity, it is implanted in the endometrium; that is, the embryo is injected to complete the pregnancy [14]. Thus, successful conception requires sperms auspiciously reaching the cervix, sperms-ova meet-up in the fallopian tubes, unhindered fertilization, successful traveling of the zygote into the uterine cavity, and successful embryo implantation. Female infertility can be caused due to the following reasons.

### 2.1. Abnormal Cervical Mucus

Abnormal cervical mucus will affect the penetration of sperm [15], making it much more difficult for them to enter the cervical opening. Under physiological conditions, cervical mucus can prevent pathogenic microorganisms from entering the uterus and infecting the endometrium [16], thus making it naturally viscous. During ovulation, to facilitate sperm entering the uterus, mucus permeability is selectively regulated under the biochemical interaction of a series of proteins and molecules [17, 18], primarily the expression levels of the trefoil factor family (TFF) peptide [15], resulting in reduced viscosity of the cervical mucus [19, 20]. This process is highly dependent on the regulation of sex hormones [21], so cervical mucus at different periods of the menstrual cycle has different mucin concentrations, which is the main reason why cervical mucus becomes thinner during ovulation [22]. The TFF is a polypeptide containing the P domain, which maintains the mucosal barrier. There are three types of human TFF, that is, TFF1, TFF2, and TFF3. TFF3 is secreted by gelatin forming mucin (GFM) cells that produce mucin [23]. It has been shown that TFF expression changes with the menstrual cycle, where the expression of TFF1 and TFF2 decreases during the ovulation period, while the expression of TFF3 significantly increases [24].

Cervical inflammation caused by pathogenic microorganism infection can also cause abnormal cervical mucus. Moreover, due to the infiltration of inflammatory secretions, patients often show sweeping changes in the amount, color, and quality of secretions [25]. At the same time, pathogens of reproductive tract infection like *Chlamydia trachomatis* and Neisseria gonorrhoeae [26, 27] are usually transmitted through sexual intercourse, which can directly lead to infertility by affecting sperm motility and impeding sperm entry.

### 2.2. Oocyte Quality

Oocyte quality is an independent factor in successful pregnancy [28, 29]. Each follicle comprises an oocyte with encapsulated granulosa cells and follicular membrane cells [30]. The average development and maturation of oocytes depend on the “nutrients” provided by granulosa cells and theca cells, such as steroid hormones, growth factors, and cytokines [31]. Studies have shown that mitochondria in granulosa cells are the core of steroid hormones required for follicular development [32]. Degraded granulosa cells are associated with mitochondrial swelling, the leading cause of oocyte apoptosis and follicular atresia [33]. Abnormal follicular development is not conducive to fertilization, fertilized egg implantation, and embryonic development [34]. Relative to it, the diseases leading to infertility mainly include POI and, more seriously, premature ovarian failure (POF) [35].

Increasing age will inevitably lead to ovaries aging [36], causing a gradual decrease in the number of follicular cells as well as the follicular pool in females, resulting in a decline in levels of inhibin B (INH-B) and anti-Müllerian hormone (AMH) secreted by granulosa cells in follicles [37], which are indicative of the declining function of ovaries, resulting in a reduction in the responsiveness of follicles to reproductive hormones [5]. “Fewer available follicles” and “decreased ovarian secretion function” are irreversible factors that contribute to female infertility [38].

In addition, bad living habits can also affect the quality of follicles by disrupting the average metabolic level [39], which is also the main reason for the gradual younger onset of POI/POF. For example, Zhang et al. [40] reported that women with BMI >29 kg/m^2^ showed lower fertility due to adverse effects of inferior follicular development on oocyte quality. Similarly, spicy food, improper sleep, and mental stress cause chronic inflammation in the body [41, 42], which result in reactive oxygen species (ROS) production and accumulation in granulosa cells to induce oxidative stress [43], which will further damage the function of organelles such as granulosa mitochondria and endoplasmic reticulum [44, 45], thus impairing the fertilization ability and normal development of oocytes [46], thus leading to infertility and adverse pregnancy outcomes. Similarly, the inflammatory-induced macrophage infiltration and significant secretion of proinflammatory factors increase the incidence of ovarian fibrosis [47–49], which compromises the ova's normal development and destroys the ovary's secretory function.

### 2.3. Ovulatory Dysfunction

Ovulatory dysfunction is the leading cause of infertility. The hypothalamic-pituitary-ovary (HPO) axis is essential in controlling female reproduction and the key to timely ovulation [50, 51]. World Health Organization (WHO) divides ovulatory dysfunction into three categories [52]: type I is gonadotropin-induced hypogonadism, mainly including hypothalamus and pituitary dysfunction, accounting for about 10% of ovulatory dysfunction; type II is HPO axis dysfunction, often due to some endocrine diseases, such as polycystic ovary syndrome (PCOS) and obesity; and type III is ovarian insufficiency. Ovulatory dysfunction mainly includes irregular ovulation and nonovulation, and such patients often presented with menstrual thinning or amenorrhea [53]. Hence, female infertility caused by ovulatory dysfunction often suggests a disordered reproductive hormone balance in patients.

PCOS is the most common ovulatory dysfunctional disease in women, accounting for approximately 80% of anovulatory infertility [54]. Research statistics show that PCOS affects 7 to 10% of women of childbearing age [55]. In recent years, it has been reported to be an endocrine disease caused by genetic, endocrine, and environmental factors [56]. Furthermore, abnormal metabolism results in persistently “high luteinizing hormone (LH)” status in patients, resulting in ovulatory dysfunction. Lifestyle adjustment is the first-line treatment for PCOS [53]. Therefore, a healthy lifestyle is essential for adjusting endocrine metabolism. In addition, Chavarro et al. [57] showed that following a nutritional diet plan benefits female fertility. Therefore, most cases of female infertility caused by ovulatory dysfunction can be prevented by changing diet and lifestyle.

Hyperthyroid hormones, caused by hyperprolactinemia (HPRL) and hypothyroidism, can interfere with the pulsed secretion of gonadotropin-releasing hormone, hinder the normal feedback regulation of HPO axis, and lead to ovulatory dysfunction. High thyroid-stimulating hormone (TSH) status induced by hyperprolactinemia and hypothyroidism can interfere with the pulsed secretion of GnRH and hinder the normal feedback regulation of the HPO axis, leading to ovulatory dysfunction [53, 58]. Furthermore, hypothalamic-pituitary failure (HPF) directly results in GnRH and/or gonadotropin (Gn) deficiency like idiopathic gonadotropic hypogonadism (IGH), panhypopituitarism, and Langerhans cell histiocytosis [50, 59].

Psychological stress-induced ovulation disorder infertility has received extensive attention in recent years. A series of neuroendocrine signal transduction produced by psychological stress will eventually be manifested as the continuous activation of the hypothalamus-pituitary-adrenal gland (HPA) axis [60], translating into the reduced release of central GnRH [61], disrupting the menstrual cycle, and inhibiting ovulation. Chronic stress directly acts on the hypothalamus to produce more corticotropin-releasing hormone (CRH) [62], while activation of the HPA axis results in more cortisol. Bolt's study has shown that cortisol and estradiol have the same coactivator to “fine-tune” transcription [63], and there is a significant overlap between glucocorticoids and estrogen-controlled signaling molecular networks [64], which indicates that elevated glucocorticoids will antagonize estrogen effects and disrupt regular ovulation. In a randomized controlled trial by Michopoulos [65], ovulation resumed in six of eight women treated with cognitive-behavioral therapy (CBT).

### 2.4. Tubal Obstruction

The anatomical-based tubal obstruction will directly hinder the sperm and egg combination, causing fertilization to fail. According to statistics, about 30% of the world's infertile women have tubal lesions [66]. Moreover, other common pathogenic contributing factors are Neisseria gonorrhoeae, *Chlamydia trachomatis*, endometriosis, and surgery [26, 67], leading to tubal infertility. Cilia in the fallopian tube become active during ovulation to transport the fertilized egg. However, pathological conditions such as tubal inflammation and hydrosalpinx result in cilia destruction, thereby reducing the ciliary movement [68], thus preventing the ova and sperm combination for successful fertilization and increasing the risk of infertility or ectopic pregnancy.

### 2.5. Endometrial Damage

Embryo implantation is the result of the interaction between blastocyst and endometrium. The key to its success lies in embryo quality and endometrium conditions. This process cannot be avoided even with assisted reproductive technology, so a good endometrium is necessary for a successful pregnancy. Endometrial receptivity (ER) is commonly used to evaluate the ability of an embryo's endometrial receptivity [69] and is closely related to the time of embryo implantation [70]. In most women, the endometrial implantation window is approximately five to seven days after ovulation [71]. Still, various pathological factors will shorten or shift the implantation window, which is not conducive to embryo implantation.

CE is a significant factor that damages the normal function and is often neglected due to the lack of apparent clinical manifestations [72]. Various “stimuli” promote changes in the number of white blood cells, cytokine production, and growth factors in the endometrial microenvironment [73], such as plasma cell infiltration and tissue edema [74], thus exacerbating their adverse effects on ER. In addition, the endometrium is regularly subjected to sex hormones under the regulation of the HPO axis, resulting in periodic growth changes. This growth pattern of the endometrium is of pivotal importance for a successful pregnancy, which CE compromises. Studies [73, 75] showed that antiapoptotic expressions, such as estrogen receptor, progesterone receptor, Ki-67 cell proliferation marker, B-cell lymphoma-2 (BCL-2), and BCL-2-associated *X* (BAX), were increased in endometrial epithelial cells and stroma of CE patients, leading to endometrial polyps and endometriosis [76]. Thus, it can be concluded that the immune disorder in the endometrial microenvironment is an essential factor leading to endometrial lesions. Endometrial polyps, endometriosis, adenomyosis, fibroids, and other space-occupying lesions can directly damage the endometrium and hinder embryo implantation. Surgical resection is the preferred treatment [77], but as an intrauterine operation, surgery has the possibility of compromising fertility, such as intrauterine adhesions [78].

In addition, CE has also been found to change the pattern of uterine contractions during ovulation and the luteal phase [79]. Under physiological conditions, in the proliferative phase, the uterus tends to contract from the fundus to the cervix, which is beneficial for menstrual discharging; in the ovulation and luteal phase, the retrograde contraction from the cervix to the fundus of the uterus is the primary process, which is conducive to the migration of sperm to the fallopian tube. However, CE reduces the probability of retrograde contractions during ovulation and the luteal phase by 3.3 folds [80], which will reduce the likelihood of successful pregnancy. It is also associated with additional discomfort symptoms, such as dysmenorrhea and pelvic pain [72, 81].

## 3. Acupuncture

Acupuncture is regarded as a multidimensional procedure that can prove being helpful in treating many diseases with minimal invasiveness using needles. It has been practiced for thousands of years, yet scientists started investigating its effects after the 18th century [82]. With the increasing application of acupuncture in clinical practice, researchers also developed a strong aptitude for researching acupuncture to treat various ailments. After decades of clinical practice and development, acupuncture was reported to possess significant clinical effects [11]. During early times, acupuncture was only realized through doctors' manipulations [83], which had high requirements for doctors' acupuncture skills. With the development of science and technology and the continuous integration of modern technology and medical technology, various acupuncture-derived therapies were introduced to strengthen the effect of acupuncture and facilitate clinical treatment, like EA and ACE.

### 3.1. Traditional Acupuncture

Traditional acupuncture involves inserting needles into meridians and acupoints [12]. To enhance the sense of needling, doctors often use auxiliary manipulation after needling the skin, such as repeatedly lifting and inserting and rotating the needling back and forth [83]. Primary scientific studies have shown [84] that manual stimulation of acupuncture needles can activate muscle afferent nerves on the one hand and exert its effect by locally generating electrical signals on the other. Manually operated acupuncture needles effectively regulate peripheral and central neural pathway activity [85]. When acupuncture is inserted into specific parts, the conduction through meridians will promote the coordination and balance of blood and energy throughout the body, producing a series of physio-psychological reactions [86, 87]. However, the manual operation of traditional acupuncture has high requirements on the physical strength of the doctor. Therefore, after inserting the needle into the corresponding acupoint, the doctor often uses electricity to translate the acupuncture into a more obvious therapeutic effect.

### 3.2. EA

EA comprises stimulating the hand-inserted needles with microcurrent waves (including continuous waves and intermittent waves), which can enhance the effect of acupuncture [88]. Furthermore, neural signals generated by EA stimulation were found to cause the hypothalamus to release endogenous opioids [89], such as *β*-endorphins, which are thought to play an essential role in regulating the effects of stress on reproductive function [90]. Previous studies have shown that [91, 92] acupuncture can change the level of plasma *β*-endorphin, thereby affecting the secretion of GnRH and Gn and then regulating the HPO axis to control female reproduction. Moreover, Stener [92, 93] reported that repeated EA therapy could reduce the high pulsatility index (PI) value in women's uterine arteries to an average level, which produced beneficial effects in increasing ER. Similarly, it can also improve the phenomenon of anovulation in PCOS patients.

Kim and Bae [94] showed that EA could produce a balance that enhanced the NK cell activity and promoted Th1/Th2 cell reaction. Moreover, Li et al. [95] demonstrated that acupuncture could inhibit free radicals (FR) metabolic imbalance and thus help achieve an antioxidant stress effect, which shows that acupuncture can regulate immunity and antioxidation, which can help regulate the immune balance in the endometrial microenvironment, treat CE, and increase ER.

### 3.3. ACE

ACE therapy is to embed absorbable sutures into acupoints, which will continuously stimulate the embedded part, to achieve the purpose of disease treatment, health care, and body strengthening [96]. The effect of catgut embedding is like that of acupuncture, but it is more lasting than acupuncture, and its stimulation can be maintained for two weeks or even longer [97]. A randomized controlled trial (RCT) conducted by Qin et al. [98] showed that ACE as a complementary therapy was beneficial for improving the rate of regular ovulation and clinical pregnancy.

## 4. Acupuncture and Infertility

### 4.1. Clinical Research

Female infertility results from an abnormal reproductive endocrine function [99]. Many diseases lead to female infertility, hindering the process of pregnancy from various nodes. Because acupuncture has the function of adjusting the neuroendocrine system [100], its application in the field of reproduction has attracted extensive attention. Acupuncture can act on multiple parts of the female reproductive system to improve its function through the action of neuroendocrine signaling molecules, to improve female fertility. Currently, acupuncture is mainly applied as a clinical adjuvant treatment of infertility conditions, such as IVF-ET and PCOS, as shown in Table 1.

Six RCTs [101–106] of IVF-ET patients treated with acupuncture showed a significantly increased clinical pregnancy rate than those without acupuncture. However, four other studies [107–110] reported the opposite results. Following a thorough analysis, we found that the RCTs that showed increased pregnancy rates were mainly from the last two to three years, while the RCTs that showed adverse effects were more than a decade old. Thus, it can be hypothesized that this could be due to the continuous development of acupuncture technology over time, which also improved the clinical efficacy of acupuncture.

Rashidi et al. [109] showed that acupuncture could improve the rate of high-quality embryos in IVF patients. Chen and Hau [110] showed that acupuncture could increase the estradiol (E2) and progesterone (P) levels in IVF patients and promote the endometrial artery blood flow; all of these are conducive to embryo transfer. Similarly, after follow-up, three studies showed significant differences in the rate of persistent pregnancy between the two groups [104–106]. Guven et al. [106] showed that IVF-ET patients treated with acupuncture had a higher live birth rate and a lower state-trait anxiety inventory-1 (STAI-1) score. Wang et al. [102] demonstrated that acupuncture could improve the endometrial morphology and menstruation in IVF-ET patients, and Zhou et al. [103] showed that acupuncture significantly improved blood E2 levels, the number of ova obtained, and the number of high-quality embryos in IVF patients.

Furthermore, Altutunji et al. [104] showed that acupuncture could increase blood E2 and P levels and reduce the incidence of ovarian hyperstimulation syndrome (OHSS). Therefore, it can be found that acupuncture can improve the clinical pregnancy rate of IVF-ET patients by ameliorating the level of sex hormones and promoting the endometrial condition. In addition, acupuncture also reduced the occurrence of ovarian hyperstimulation syndrome (OHSS) and alleviated patients' anxiety to a certain extent.

Three other RCTs [111–113] reported the effect of EA on IVF-ET infertility patients. Kusuma et al. [111] showed that EA could improve the number of ova obtained by IVF. Further testing found that BAX expression decreased, and BCL-2 expression increased in patients with EA treatment, which confirmed that EA could help patients get more follicles by inhibiting granulosa cell apoptosis. However, Wu et al. [112] and Xiang et al. [113] showed opposite results regarding the number of obtained ova but concluded that EA could significantly improve the rate of high-quality embryos in IVF patients. However, their research results on clinical pregnancy rates were different. We speculate that this may be related to the course of EA treatment. Studies with longer EA treatment cycles have shown better efficacy in clinical pregnancy rates than short-term EA treatment [112]. The study of Xiang et al. [113] showed that EA could significantly improve the live birth rate of IVF patients, although there was no significant difference in clinical pregnancy rate. Therefore, we can find that EA can enhance ova quality to a certain extent, but further facilitating the pregnancy outcome may require a long period of repeated EA stimulation.

Three other RCTs [114–116] reported the effect of TEAS on patients with IVF-ET infertility. Qu et al. [114] and Shuai et al. [116] reported that TEAS significantly increased the clinical pregnancy rate and live birth rate in IVF patients compared with those without TEAS intervention. Similarly, Zhai et al. [115] showed that TEAS (20/30/40 mA) showed no significant difference in clinical pregnancy rate compared to TEAS (5 mA), depicting that though TEAS is beneficial for pregnancy outcomes, in IVF-ET patients, the optimal stimulation intensity of TEAS is yet to be explored.

Four RCTs [117–120] investigated the effect of acupuncture on infertility patients with PCOS. Jiang et al. [117] and Xu et al. [119] reported that the group with acupuncture intervention had a significant increase in clinical pregnancy rate compared to the group that received only western medicine treatment regimen. However, Jiang and Xu's findings contradicted the study conducted by Yu et al. [120]. Moreover, it was reported that acupuncture can improve the cycle ovulation rate, E2 and P levels, and endometrial morphology is also envisaged to benefit patients with PCOS. Xu et al. [119] also reported that acupuncture could improve the rate of regular ovulation and reduce serum *T* and LH levels in infertility patients with PCOS. Nevertheless, Wu et al. [118] reported that acupuncture could not improve the live birth rate. Therefore, it is hypothesized that acupuncture could help PCOS patients ovulate by improving sex hormone levels before pregnancy, thus increasing the pregnancy rates. However, the therapeutic effects of acupuncture before pregnancy may not last until delivery.

### 4.2. Animal Studies

The detailed information regarding acupuncture in animals is shown in Table 2. Stener-Victorin reported that repeated EA stimulation significantly promoted the release of *β*-endorphins in the hypothalamus of polycystic ovary (PCO) rats and reduced nerve growth factor (NGF), corticotropin-releasing factor (CRF), and endothelin-1 (ET-1) in the ovaries of PCO rats [95, 121–123]. The *β*-endorphins can inhibit GnRH secreted by the hypothalamus and LH released by the pituitary [124]. Some scholars argue that endogenous opioid drugs are closely related to the surge of LH before ovulation [125, 126]. Therefore, EA helps improve the “high-LH” state and restore normal ovulation function for PCO rats. The increase in nerve growth factor (NGF) and endothelin-1 (ET-1) was found to be associated with ovarian sympathetic excitation [127, 128], which has been reported in many inflammatory and autoimmune states [129]. The NGF is one of the target neurotrophic factors involved in developing and maintaining ovarian innervation [130]; ET-1 is a vital peptide that regulates blood flow in the ovary and is an effective and durable vasoconstrictor [122]. CRF is related to stress [131]. The repeated EA treatment was also found to improve the frequency and activation of *T* and natural killer (NK) cells, but the difference was insignificant.

Similarly, 12 cycles of EA treatment did not significantly improve ovarian morphology. However, it substantially improved the ovarian neuroendocrine function in PCO rats. The authors speculated that more extended periods of EA might translate into significant effectiveness. Zhang [132] demonstrated that acupuncture could significantly downregulate serum testosterone (*T*) and upregulate E2 expression in PCO rats, improve ovarian function, promote endometrial development, and promote embryo implantation.

Huang et al. [133] reported that EA could reduce serum *T*, LH, and AMH contents, reduce the ratio of ovarian LC3-II/I, and upregulate phosphatidylinositol-3-kinase (PI3K) and protein kinase B (PKB, also known as AKT) in PCO rats. The LC3 is a biomarker of autophagy. Cytoplasmic LC3 (LC3-I) will hydrolyze a small peptide and transform it into autophagosome (LC3-II), representing a direct relationship between a higher LC3-II/I ratio and a higher the level of autophagy.

A reduction in ovarian reserve function directly affects female reproduction ability. An increase in FSH and a decrease in E2 levels are typical of decreased ovarian reserve function [134]. Follicular development and maturation result from the oocytes' coregulation, mutual influence, and surrounding granule cells. It has been found that granulosa cells provide nutrients and growth signals for oocytes, and their apoptosis is the primary reason for follicular atresia [135]. A hormone is an important signal molecule in granulosa cell proliferation and apoptosis. In ovarian dysfunction, the sensitivity of follicles to hormones reduces and declines the ovaries' secretary function for estrogen and progesterone [136], both of which are not conducive to follicular development. FSH is an essential hormone for follicular development, which can bind to the FSH receptor on the granular cell membrane to activate upstream protein kinase A (PKA) and Grb2-associated Binder2 (GAB2), and downstream target factors and PI3K/AKT pathway are then activated to slow down the apoptosis of granulosa cells [137, 138]. Zhao et al. [139] showed that repeated EA stimulation significantly increased blood E2 concentration and restored HPO axis function in ovariectomy (OVX) rats. Further analysis showed that EA increased aromatase activity, mRNA, and protein expression in OVX rats, suggesting that FSH can also induce aromatase expression, stimulate ovarian E2 secretion, and promote granulosa cell maturation [136].

Wang et al. [140] showed that manual acupuncture could regulate hormone levels in POF rats (increase E2 and decrease FSH), upregulate PI3K/AKT signaling pathway, and promote follicular development, where higher expressions of PI3K, AKT, BCL-2 gene, and proteins were observed. In contrast, the expression of BAX decreased in POF rats after manual acupuncture, which could help reduce apoptosis of granulosa cells and reduce follicular atresia. In terms of morphology, though, acupuncture did not significantly reduce the apoptosis of granulosa cells in POF rats, suggesting that acupuncture was more about improving ovarian function. However, Zhang et al. [141] reported that EA reduced the phosphorylation of PI3K, AKT, mammalian target of rapamycin (mTOR), S6 kinase (S6K), and 4E-binding protein 1 (4E-BP1) and downregulated the ovarian PI3K/AKT/mTOR activation pathway in POF mouse. In terms of hormone levels, EA can upregulate serum AMH and E2 in POF mice and downregulate serum FSH and LH levels, which agrees with the reports of other researchers; hence, acupuncture is speculated to be beneficial to the level of sex hormones in POF rats.

Female POF mice treated with EA mated with male mice, and the outcome was compared with mice not subjected to EA treatment [141]. The results indicated that the EA group's litter size was significantly increased, indicating that acupuncture can improve the fertility of POF mice. Gao et al. [142] used mifepristone in pregnant rats to establish an “embryo implantation failure model.” After manual acupuncture treatment, compared with the nonacupuncture group, the number of implanted embryos, mRNA, and protein levels of CCL2 (CC chemokine subfamily L2) and CXCL8 (CXC chemokine subfamily L8) in the endometrium and uterine NK (uNK) cell subpopulations were significantly higher. The CCL2, CXCL8, and uNK cells are closely related to placental development [143]. The CCL2 can promote Th2 polarization and maintain a Th2 dominant environment, thus ensuring embryo implantation by regulating immunity [144]; CXCL8, on the other hand, stimulates the invasion of trophoblast cells outside villus in early pregnancy into the decidua by increasing MMP-2 secretion [145]. However, uNK cells in rats only appear during pregnancy. They often promote angiogenesis by expressing various cytokines, such as vascular endothelial growth factor (VEGF), placental growth factor (PGF), and angiopoietin 2 (ANG2), which is conducive to trophoblast invasion and placenta formation [146, 147]. This experiment suggested that acupuncture helps regulate the endometrial microenvironment through cytokine and chemokine pathways to aid embryo implantation during pregnancy. Zhu et al. [148] also reported that repeated EA stimulation could increase the secretion of insulin growth fact-1 (IGF-1) in the endometrium, thus improving the embryo implantation rate in mice. Fu et al. [149] reported that acupuncture could reduce the higher level of E2 in superovulation rats, and further studies found that the expression of estrogen receptor -*β* increased in rats' pituitary. These results suggest that acupuncture can prevent and reduce the incidence of OHSS by reducing the excessive increase in serum E2, which reflects the bidirectional adjustment ability of acupuncture and high safety.

## 5. Mechanism of Acupuncture Treatment of Female Infertility

As previously described, acupuncture has a positive treatment effect on female infertility. However, the causes of infertility vary, and understanding the role of acupuncture will help apply it to the appropriate type of infertility to achieve maximum efficacy. Based on the existing studies, it was found that acupuncture is beneficial in regulating female reproductive hormones and various cellular and immune signaling molecules, which are considered helpful in improving multiple aspects of the female reproductive system, such as follicular development, regular ovulation, and embryo implantation. Therefore, acupuncture has great application value in PCOS, POI, and IVF-ET. Furthermore, as a complementary and alternative therapy, acupuncture can improve female fertility and the success rate of assisted reproductive technology. As shown in Figure 1, the therapeutic effect of acupuncture on female infertility is mainly aimed at the following three aspects: reproductive endocrine, follicular development, and embryo implantation. The various mechanistic implications of acupuncture therapy in female infertility are discussed below.

### 5.1. Reproductive Endocrine Pathway

The reproductive hormones are at their basic level during the follicular phase, and withdrawal of estrogen and progesterone induces menstruation. Low levels of E2 and P will alternatively promote the secretion of GnRH, encouraging the secretion of Gn (FSH and LH), which is essential for follicles development and results in the secretion of E2 and P. E2 and P are the material basis of endometrial proliferation and transformation and facilitate it in accepting embryos. This serial effect ensures the synchronization of follicular development and endometrial development required for pregnancy. The basic endocrine level of infertile women is “high Gn,” which inhibits follicular growth since higher levels of Gn inhibit the secretion of E2 and P, resulting in no longer regular ovulation, leading to infertility. Acupuncture can restore normal reproductive hormone levels. While reducing GnRH, FSH, LH, and increasing E2 and P, it is more important to restore the regularity of hormone interaction, make the reproductive system usually operate, and then promote pregnancy.

### 5.2. Improvement in Ovarian Function

There are two main ways to improve ovarian function: reducing granulosa cell apoptosis in follicles and improving the ovarian environment. During follicular development, granulosa cells are responsible for providing nutrients required maturation of the ovum. Follicular atresia and apoptosis are closely related to granulosa cell apoptosis. Acupuncture can increase the expression of BCL-2 and reduce the expression of BAX to reduce the apoptosis of granulosa cells, hence serving as an escort for follicular development. On the other hand, the internal ovarian environment is a prerequisite for follicular development. Acupuncture can reduce the expression of NGF, CRF, and ET-1 to reduce inflammation in the ovary and promote the blood supply in the ovary.

### 5.3. Improvement in Embryo Implantation

The interaction of an embryo with the endometrium microenvironment to form a biological connection refers to embryo implantation. Acupuncture can promote embryo implantation by three mechanisms, that is, modulating autoimmunity, where acupuncture resists the maternal immune response to embryos (foreign objects) by increasing the expression of CCL2. Similarly, by increasing the expression of CXCL8 and MMP-2, trophoblast cells can invade decidual tissue to establish a physical connection with the endometrium. The second mechanism refers to feeding, where acupuncture increases the expression of VEGF, ANG2, and PGF to promote angiogenesis, to establish the pathway of material exchange between mother and embryo. Finally, the other mechanism embarks on embryonic development, where acupuncture helps the development of embryos in the endometrium by increasing the expression of IGF-1. The classification and summary of relevant mechanisms are shown in Figure 2.

## 6. Summary and Outlook

The etiology of female infertility is complex and can be multifactorial, that is, pathological, physiological, psychological, and social. This review discusses the incidence of female infertility during the whole pregnancy cycle for the first time, which is envisaged to help understand the causes of female infertility and help target the clinical diagnosis and treatment. Female reproduction needs the reproductive system to provide a reasonable “material basis” on the one hand, and the neuroendocrine system to release accurate “signal” regulation on the other hand. Thus, successful pregnancy embodies the perfect cooperation between the reproductive and neuroendocrine systems. This ideal state is reflected in the interaction between signal molecules to achieve “dynamic balance.” A good “material base” is necessary for follicular development and endometrial growth.

Initially, the HPO axis is in a positive activation state: the hypothalamus releases GnRH, which prompts the pituitary gland to release FSH and LH, and the ovary begins to produce E2. Simultaneously, follicles start to develop, and intima begins to proliferate. Until the follicle maturation, LH and E2 levels significantly increase, followed by a negative activation state elicited by the HPO axis, resulting in LH and E2 levels dropping precipitously, thus inducing ovulation. Following this, the level of P rises, and the endometrium begins to prepare for embryo implantation. Hormones, as nutrients, participate in the whole process of follicular and intimal development. At the same time, its interaction precisely controls the entire process. The orderly progress of this process is the “balance state” of the female reproductive endocrine. An abnormality in any of these processes results in missing the pregnancy opportunity or might translate into unacceptable conditions for pregnancy, leading to infertility. For example, high LH will inhibit the production of E2 and P by a feedback mechanism, hindering follicular maturation, resulting in failure of endometrium transformation from proliferative to secretory phase. The key to successful pregnancy lies in the regular appearance of specific signal molecules and the “steady state” of the body's internal environment.

Based on existing studies, it was observed that the mechanism of acupuncture in the treatment of infertility is mainly reflected in four ways, that is, by adjusting HPO axis balance, where acupuncture reduces the “high GnRH” and “high LH” status in PCO rats by increasing the expression of *β*-endorphins, which is beneficial to follicular development. The second mechanism involves improving the ovary's internal environment by increasing ovarian blood flow and reducing the ovary's immune-inflammatory response by decreasing the expression of NGF, CRF, and ET-1. The third mechanism involves increasing the expression of BCL-2 and decreasing the expression of BAX and LC3-II to LC3-I ratio to reduce granulosa cell apoptosis and promote T's transformation to E2 by activating aromatase. The final mechanism involves helping the embryo implantation by upregulating the expression of IGF-1, CCL2, and CXCL8 signaling molecules to promote placental growth and ensure embryo implantation. All these mechanisms are conducive to restoring women's normal reproductive hormone levels, improving the function of the female reproductive system, and promoting the occurrence of pregnancy. The event of infertility is often the result of an “imbalance” in the human internal environment, such as “high GnRH” and “high LH.” Therefore, acupuncture can comprehensively regulate various signal molecules in the human body and improve reproductive function from multiple angles. Based on the above studies, it is believed that acupuncture as a complementary and alternative therapy in assisted reproduction could be meaningful.

Acupuncture has also been widely used in clinics, where in addition to its curative effect, its simple operation and fewer adverse reactions are additional advantages. Different from the endogenous reaction caused by drugs, as a surgical operation, acupuncture treatment does not involve the use of any chemicals; hence, it is considered relatively safe. At present, the current research results are not entirely consistent. We speculate that it is mainly due to clinical heterogeneity, including different acupuncture schemes and doctors' levels. Although acupuncture is easy to operate, its efficacy is determined by the angle, depth, single duration, optimal acupuncture time, treatment course of acupuncture, different acupuncture manipulations at different acupoints, and differences in individual responsiveness of patients. Differences in these control variables lead to heterogeneity between clinical studies and are the main reason for the inconsistent research results, yet the effectiveness of acupuncture cannot be ignored. Based on the existing clinical reports, we can find that the positive effect of acupuncture was reflected in all aspects conducive to pregnancy, as shown in Table 3. We can divide these evaluation indicators into two categories: prepregnancy indicators (detection indicators), which are the conditions to increase the probability of pregnancy, while the other is the observation index after pregnancy (i.e., to observe the pregnancy outcome intuitively). The reports on negative results only focused on the observation indicators after pregnancy, that is, pregnancy outcome. However, the positive effects of acupuncture on the physical state of infertile women were never denied. We know that exploring the differences in pregnancy outcomes is more challenging than detecting indicators with more stringent requirements in research design and observation duration. The premise of pregnancy is to have a good physical state. It mainly refers to mature follicles, high-quality embryos, and good endometrium, necessary conditions for a successful pregnancy. Therefore, in the process of observation and research, the effectiveness of acupuncture may first be reflected in the above aspects, followed by pregnancy outcomes. Thus, acupuncture is believed to be equally effective in resolving infertility issues through comprehensive analysis. It also necessitates studying the effectiveness of acupuncture in treating females' infertility by comparing results from different treatment cycles among other patient groups. It is believed that acupuncture effectiveness can be significantly reflected in longer treatment cycles, also reflected in the current research results, which are envisaged to help a more comprehensive understanding of acupuncture, improving the overall physiological function of infertile women.

Therefore, optimizing the acupuncture treatment plan in an all-around way will improve the clinical curative effect and help us explore acupuncture deeply. Similarly, it is suggested that more rigorous and more targeted studies in the future may provide strong evidence and help determine the application suitability of acupuncture in the field of reproduction, making it worthy of further investigation.

## 7. Conclusion

Acupuncture and related therapy can restore the average balance and regularity of sex hormones in infertile women by decreasing serum FSH and LH levels and increasing E2 and P levels, which are beneficial for follicle development and maturation, regular ovulation, and the normal physiological function of the inner membrane, which is conducive to conception. As a complementary and alternative therapy, acupuncture can play a positive role in PCOS-infertility, POI- infertility, and IVF-ET, with clinical application value.

## Figures and Tables

**Figure 1:** Mechanism of acupuncture in the treatment of infertility. The main function of acupuncture is to regulate reproductive related neuroendocrine signal molecules, in order to balance female reproductive endocrine, improve ovarian function, and promote embryo implantation. The symbol “⬆” represents increased expression and activity of the molecule, and the symbol “⬇” represents a decrease in the expression of this molecule. The symbol “+” represents positive feedback regulation, and the symbol “−” represents negative feedback regulation. Abbreviations are listed at the end of the article.

**Figure 2:** Classification of the mechanisms of acupuncture in treating infertility. The symbol “⬆” represents increased expression and activity of the molecule, and the symbol “⬇” represents a decrease in the expression of this molecule.

**Table 1:** Characteristics of clinical studies.

First author	Year	Research type	Type of infertility	Intervention		Course of treatment	Evaluating indicator	
				*T*	*C*		*P* < 0.05	*P* > 0.05
Andersen D	2010	RCT	IVF-ET	Acupuncture	N	1 time	——	CPR, PPR, LBR (−)
Moy I	2010	RCT	IVF-ET	Acupuncture	N	1 time	——	CPR (−)
Rashidi BH	2013	RCT	IVF-ET	Acupuncture	N	4 times	NHQE⬆	NRO, CPR, PPR, BPR (−)
Villahermosa DI	2013	RCT	IVF-ET	Acupuncture	N	4 times	CPR⬆	——
Chen Q	2015	RCT	IVF-ET	Acupuncture	N	12 weeks	(E_2_, P)⬆, EAI⬇	CPR (−)
Jiang D	2015	RCT	PCOS	Acupuncture + WM	WM	12 weeks	(CPR, ET/EM, CM)⬆, AR⬇	——
Wang X	2016	RCT	IVF-ET	Acupuncture	N	30 times	(CPR, EM, Menstruation)⬆	——
Zhou L	2016	RCT	IVF-ET	Acupuncture	N	15 ± 2 times	(E_2_, NRO, NHQE, CPR)⬆	——
Qu F	2017	RCT	IVF-ET	TEAS	N	2 times	(CPR, LBR, NPY)⬆	NRO, FR, NHQE, TGF-*α*, G-CSF (−)
Wu XK	2017	RCT	PCOS	Acupuncture + WM	WM	16 weeks	——	LBR (−)
Xu J	2018	RCT	PCOS	Acupuncture + WM	WM	8 weeks	(CPR, COR)⬆, (T, LH)⬇	AR, ET (−)
Yu L	2018	RCT	PCOS	Acupuncture + WM	WM	24 times	(COR, ET/EM, E_2_, P)⬆	CPR (−)
Altutunji AZ	2019	RCT	IVF-ET	Acupuncture	N	2 weeks	(CPR, PPR, E_2_, P)⬆, OHSS incidence⬇	AMH (−)
Kusuma AC	2019	RCT	IVF-ET	EA	False EA	6 times	(NRO, FR, BCL-2)⬆, BAX⬇	GDF9, BMP15 (−)
Shuai Z	2019	RCT	IVF-ET	TEAS	N	16 ± 2 times	(CPR, LBR)⬆	——
Wu HC	2019	RCT	IVF-ET	EA	False EA	12 weeks	(NHQE, CPR, PI3K/Akt mRNA)⬆	NRO (−)
Dehghani AS	2020	RCT	IVF-ET	Acupuncture	N	2 times	(CPR, PPR)⬆, BPR⬇	——
Guven PG	2020	RCT	IVF-ET	Acupuncture	N	3 times	(CPR, PPR, LBR)⬆, STAI-1 score⬇	——
Xiang S	2021	RCT	IVF-ET	EA	N	24 times	(NHQE, LBR, IRS-1/PI3K/GLUT4 mRNA)⬆	NRO, CPR (−)
Zhai ZJ	2021	RCT	IVF-ET	TEAS (20 mA/30 mA/40 mA)	TEAS (5 mA)	10–13 times	(NRO, ET)⬆	NHQE, CPR (−)

*Note.* T: Test group; C: Control group; RCT: Randomized controlled trial; IVF-ET: In vitro fertilization - embryo transfer; PCOS: Polycystic ovary syndrome; EA: Electroacupuncture; TEAS: Transcutaneous electrical acupoint stimulation; N: None; WM: Western medicine; CPR: Clinical pregnancy rate; PPR: Persistent pregnancy rate; LBR: live birth rate; BPR: Biochemical pregnancy rate; COR: Cycle ovulation rate; AR: Abortion rate; FR: Fertilization rate; NRO: Number of retrieved oocytes; NHQE: Number of high-quality embryos; ET: Endometrial thickness; EM: Endometrial morphology; EAI: Endometrial arterial impedance; CM: Cervical mucus; E_2_: Estradiol; P: Progesterone; STAI-1: State-trait anxiety inventory-1; OHSS: Ovarian hyperstimulation syndrome; NPY: Neuropeptide Y; TGF-*α*: Transforming growth factor-*α*; G-CSF: Granulocyte colony stimulating factor; BCL-2: B-cell lymphoma-2; BAX: Bcl2-Associated X; PI3K: Phosphatidylinositol-3-kinase; AKT: Protein kinase B; IRS-1: Insulin receptor substrate-1; GLUT4: Glucose transporter 4; GDF9: Growth differentiation factor 9; BMP15: Bone morphogenetic protein 15; ⬆: Improve; ⬇: Reduce; (−): Unchanged.

**Table 2:** Characteristics of animal studies.

First author	Year	Experimental object	Modeling drugs	Intervention	Course of treatment (times)	Evaluating indicator	
						*P* < 0.05	*P* > 0.05
Stener-victorin E	2000	PCO rats	EV	EA	12	NGF⬇	Ovarian morphology (-)
Stener-victorin E	2001	PCO rats	EV	EA	12	CRF⬇	——
Stener-victorin E	2003	PCO rats	EV	EA	12	NGF⬇, ET-1⬇	——
Stener-victorin E	2004	PCO rats	EV	EA	12	*β*-Endorphins⬆	NK cell, CD4 + /CD8 + T cell (-)
Zhang WY	2009	PCO rats	DHEA	Acupuncture	5	(NEI, Ovarian morphology, ET, E_2_)⬆, T⬇	TSH, LH, P (-)
Huang J	2020	PCO rats	LE	EA	14	(AMH, PI3K, AKT)⬆, (T, LH, LC3 II/I)⬇	Ovarian morphology (-)
Gao W	2013	ETF rats	Mifepristone	Acupuncture	10	(NEI, CCL2, CXCL8, uNK cell subsets)⬆	——
Zhu S	2016	COH mice	Gn	EA	7	(NEI, IGF-1)⬆	——
Wang S	2019	POF rats	CTX	Acupuncture	21	(E_2_, PI3K, Akt, BCL-2)⬆, (BAX, FSH)⬇	Ovarian morphology (-)
Zhong H	2019	POF rats	CTX	EA	7	(NF, LS, E2, AMH)⬆, (PI3K, AKT, mTOR, S6K, 4E-BP1, FSH, LH)⬇	——

*Note.* PCO: Polycystic ovary; ETF: Embryo transfer failure; COH: Controlled ovarian hyperstimulation; POF: Premature ovarian failure; EV: Estradiol valerate; DHEA: Dehydroepiandrosterone; LE: Letrozole; Gn: Gonadotropin; CTX: Cyclophosphamide; EA: Electroacupuncture; NGF: Nerve growth factor; CRF: Corticotropin releasing factor; ET-1: Endothelin-1; FSH: Follicle stimulating hormone; E_2_: Estradiol; T: Testosterone; ET: Endometrial thickness; NEI: Number of embryo implantation; LH: Luteinizing hormone; AMH: Anti-Mullerian hormone; LC3: Microtubule associated protein 1 light chain 3; PI3K: Phosphatidylinositol-3-kinase; AKT: Protein kinase B; CCL2: CC chemokine subfamily L2; CXCL8: CXC chemokine subfamily L8; IGF-1: Insulin growth factor; BCL-2: B-cell lymphoma-2; BAX: Bcl2-Associated *X*; NK cell: Natural killer cell; mTOR: mammalian target of rapamycin; S6K: S6 kinase; 4E-BP1: 4E-Binding Protein1; NF: Number of follicles; LS: Litter size; ⬆: Improve; ⬇: Reduce; (-): Unchanged.

**Table 3:** Classification of clinical evaluation indexes of acupuncture in the treatment of infertility.

Evaluation category	Specific items			
*Evaluation index before pregnancy*				

Cervix	CM	⬆	——	
Endometrium	EAI, ET, EM	⬆	——	
Ovary	NRO, COR	⬆	——	
Embryo	FR, NHQE	⬆	——	
Menstruation	Menstrual regularity	⬆	——	
Ovarian function markers	NPY, AMH, BCL-2, IRS-1, (PI3K, Akt, GLUT4) mRNA	⬆	BAX	⬇
Hormone level	E_2_, P	⬆	T, LH	⬇
Security	——	OHSS incidence	⬇	

*Evaluation index after pregnancy*				
Pregnancy outcome	CPR, PPR, LBR	⬆	BPR, AR	⬇

*Note.* CM: Cervical mucus; EAI: Endometrial arterial impedance; ET: Endometrial thickness; EM: Endometrial morphology; NRO: Number of retrieved oocytes; COR: Cycle ovulation rate; FR: Fertilization rate; NHQE: Number of high-quality embryos; NPY: Neuropeptide Y; AMH: Anti-Mullerian hormone; BCL-2: B-cell lymphoma-2; IRS-1: Insulin receptor substrate-1; PI3K: Phosphatidylinositol-3-kinase; AKT: Protein kinase B; GLUT4: Glucose transporter 4; BAX: Bcl2-Associated *X*; E_2_: Estradiol; P: Progesterone; T: Testosterone; LH: Luteinizing hormone; OHSS: Ovarian hyperstimulation syndrome; CPR: Clinical pregnancy rate; PPR: Persistent pregnancy rate; LBR: live birth rate; BPR: Biochemical pregnancy rate; AR: Abortion rate; ⬆: Improve; ⬇: Reduce.

## Data Availability

The data used to support the findings of this study are included within the article.

## Abbreviations

POI: Premature ovarian insufficiency
PCOS: Polycystic ovary syndrome
CE: Chronic endometritis
AI: Artificial insemination
IVF: In vitro fertilization
IVF-ET: In vitro fertilization-embryo transfer
ICSI: Intracytoplasmic sperm injection
CAM: Complementary and alternative medicine
EA: Electroacupuncture
ACE: Acupoint catgut embedding
TEAS: Transcutaneous electrical acupoint stimulation
TFF: Trefoil factor family
GFM: Gelatin forming mucin
POF: Premature ovarian failure
INH-B: Inhibin B
AMH: Anti-Mullerian hormone
ROS: Reactive oxygen species
HPO: Hypothalamic-pituitary-ovary
LH: Luteinizing hormone
HPRL: Hyperprolactinemia
TSH: Thyroid stimulating hormone
GnRH: Gonadotropin-releasing hormone
HPF: Hypothalamic-pituitary failure
Gn: Gonadotropin
IGH: Idiopathic gonadotropic hypogonadism
HPA: Hypothalamus-pituitary-adrenal
CRH: Corticotropin releasing hormone
CBT: Cognitive behavioral therapy
ER: Endometrial receptivity
BCL-2: B-cell lymphoma-2
BAX: BCL-2-associated X
FR: Free radicals
RCT: Randomized controlled trial
E2: Estradiol
P: Progesterone
STAI-1: State-trait anxiety inventory-1
OHSS: Ovarian hyperstimulation syndrome
PCO: Polycystic ovary
NGF: Nerve growth factor
CRF: Corticotropin releasing factor
ET-1: Endothelin-1
LC: Light chain
T: Testosterone
PI3K: Phosphatidylinositol-3-kinase
PKB: Protein kinase B
PKA: Protein kinase A
GAB2: Grb2-associated Binder2
OVX: Ovariectomy
Mtor: Mammalian target of rapamycin
S6K: S6 kinase
4E-BP1: 4E-Binding Protein1
CCL2: CC chemokine subfamily L2
CXCL8: CXC chemokine subfamily L8
MMP-2: Matrix metalloproteinase-2
VEGF: Vascular endothelial growth factor
PGF: Placental growth factor
ANG2: Angiopoietin 2
IGF-1: Insulin growth fact-1
PI: Pulsatility index.
